# ETNK2 Low-Expression Predicts Poor Prognosis in Renal Cell Carcinoma with Immunosuppressive Tumor Microenvironment

**DOI:** 10.1155/2023/1743357

**Published:** 2023-02-21

**Authors:** Jian Chu, Xiong-Xian Qian, Xiang-Min Zhang, Ting Jiang, Xiao-Jun Li, Wei Sun

**Affiliations:** ^1^Department of Urology, Shanghai Baoshan Luodian Hospital, Baoshan District, Shanghai 201908, China; ^2^Department of Urology, The First People's Hospital of Taicang City, Taicang Affiliated Hospital of Soochow University, Suzhou, China

## Abstract

**Background:**

The ethanolamine kinase 2 (ETNK2) gene is implicated in carcinogenesis, but its expression and involvement in kidney renal clear cell carcinoma (KIRC) remain unknown.

**Methods:**

Initially, we conducted a pan-cancer study in which we searched the Gene Expression Profiling Interactive Analysis, the UALCAN, and the Human Protein Atlas databases to determine the expression level of the ETNK2 gene in KIRC. The Kaplan–Meier curve was then used to calculate the overall survival (OS) of KIRC patients. We then used the differentially expressed genes (DEGs) and enrichment analysis to explain the mechanism of the ETNK2 gene. Finally, the immune cell infiltration analysis was performed.

**Results:**

Although the ETNK2 gene expression was lower in KIRC tissues, the findings illustrated a link between the ETNK2 gene expression and a shorter OS time for KIRC patients. DEGs and enrichment analysis revealed that the ETNK2 gene in KIRC involved multiple metabolic pathways. Finally, the ETNK2 gene expression has been linked to several immune cell infiltrations.

**Conclusions:**

According to the findings, the ETNK2 gene plays a crucial role in tumor growth. It can potentially serve as a negative prognostic biological marker for KIRC by modifying immune infiltrating cells.

## 1. Introduction

Renal cell carcinoma (RCC) is characterized by the growth of malignant tumors within the renal tubular epithelial cells. This cancer accounts for nearly 90% of renal and 3% of all adult cancers [1]. The most prevalent kind of RCC is kidney renal clear cell carcinoma (KIRC). Due to the high prevalence of asymptomatic KIRC patients, around one-third of KIRC patients are diagnosed at an advanced stage. RCC is gaining attention because it is the third most fatal urinary system tumor, trailing only prostate and bladder cancer in terms of mortality rate [2]. Every year, nearly 430,000 new cases of RCC are diagnosed worldwide, with approximately 180,000 dying due to this disease. The incidence and mortality rates of RCC continue to rise, posing a significant risk to human health. Because of its natural resistance to chemotherapy and radiotherapy [3], the prognosis for advanced KIRC is dismal [4]. Therefore, identifying novel biological markers that aid in the early detection and treatment of this illness is critical.

Ethanolamine kinase 2 (ETNK2) is a protein-coding gene. Spondylometaphyseal dysplasia with cone-rod dystrophy is one of the diseases linked to the *ETNKT2* gene. Glycerophospholipid biosynthesis and nuclear receptor meta-pathways are two of the ETNK2-related pathways. The Gene Ontology (GO) annotations associated with this gene include ethanolamine kinase and transferase activity and the transfer of phosphorus-containing groups. The ETNK1 gene is a significant paralog of the ENTK2 gene [5]. The ETNK2 gene is associated with a poor prognosis in gastric cancer patients because it inhibits the p53-Bcl2 apoptotic pathway, which promotes liver metastasis. The ETNK2 gene has been shown to benefit phosphatidylethanolamine production in non-small-cell lung cancer significantly. In contrast, the depletion of TET2-targeted demethylation is responsible for the decreased expression of the ETNK2 gene in prostate cancer [6, 7]. Simultaneously, molecular research has revealed that the ETNK2 gene is a novel molecular marker for breast cancer (BRCA) pathogenesis [8]. The ETNK2 gene is a novel molecular marker that provides insights into the role of survival risk in several cancers. However, the function of the ETNK2 gene in KIRC has not yet been thoroughly investigated.

Moreover, the exact function of the ETNK2 gene in patients with KIRC remains unknown. Therefore, we first collected RNA-sequencing and clinical data from KIRC patients using the Cancer Genome Atlas (TCGA) datasets in this study. Following that, we discovered that ETNK2 gene expression was downregulated in KIRC patients and was linked to highly aggressive clinical and pathological characteristics. Furthermore, we investigated the diagnostic and prognostic efficacy of the ETNK2 gene in KIRC and the comprehensive relationship between the ETNK2 gene and immune characteristics. We also conducted an enrichment analysis to determine its potential signaling pathways and pathophysiological mechanisms. Finally, we used tissues from the patient's tumors and surrounding normal tissues to confirm the dysregulation of the ETNK2 gene in KIRC patients.

## 2. Materials and Methods

### 2.1. Gene Expression Analysis of the ETNK2 Gene

We obtained the study's data from the UCSC database (https://xenabrowser.net/). From the database, the unified and standardized pan-cancer dataset TCGA target Genotype-Tissue Expression (GTEX) (PanCAN, *n* = 19,131, *g*=60,499) was downloaded. Furthermore, the ETNK2 gene expression data were derived from various samples. Finally, we eliminated cancer types with fewer than 3 samples within a single cancer type, leaving 34 cancer types for which we collected expression data.

### 2.2. Survival Analysis

The patients were divided into the following two groups based on the median level of ETNK2 gene expression: the low and high-expression groups. The statistical analysis of survival data was carried out using the R software's “survival” function. The Kaplan–Meier (K–M) curves were created using the R package “survminer” to visually display the results of the survival analyses. This study investigated the prognostic significance of the ETNK2 gene expression concerning overall survival (OS) was investigated.

### 2.3. Immune Checkpoint Analysis

We extracted the expression data of the ETNK2 gene and 60 marker genes from 2 types of immune checkpoint pathway genes in each sample from the dataset. Simultaneously, we filtered all normal samples and transformed each expression value with log2 (*x* + 0.001). The Pearson correlation between the ETNK2 gene and 5 different immune pathway marker genes was then computed.

### 2.4. Analysis and Validation of the ETNK2 Gene in KIRC

We used the Gene Expression Profiling Interactive Analysis (GEPIA), a program for studying gene expression that is provided in the form of an interactive online platform, with 9,736 tumors and 8,587 normal samples from the TCGA and GTEX databases to provide additional evidence supporting the robustness of the comparison between KIRC and normal samples regarding the level of hub gene expression. Using the GEPIA platform, we also assessed the potential prognostic significance of hub genes. We calculated OS's hazard ratio (HR) and the 95% confidence intervals (CI). The K–M curve and boxplot from the TCGA database were used to visualize the relationships between gene expression and patient prognosis.

### 2.5. Identification of DEGs

The “limma” R package was used to analyze the differences in messenger RNA (mRNA) expression between the high and low ETNK2 groups. “Adjusted *P* < 0.05 and Log2 (fold change) > 1 or Log2 (fold change) < −1” were selected as the cut-off points for differentially expressed mRNAs.

### 2.6. Enrichment Analysis

The data were analyzed using functional enrichment to confirm the fundamental function of prospective targets. GO is a widely used tool for the annotation of genes with functions, particularly cellular components (CC), biological processes (BP), and molecular functions (MF). The Kyoto Encyclopedia of Genes and Genomes (KEGG) enrichment analysis is a useful tool for investigating gene functions and the high-level genomic functional data associated with those functions. The clusterProfiler tool (version: 3.18.0) in R was used to investigate the GO function of potential targets and enrich the KEGG pathway to better understand how mRNA contributes to cancer progression. The boxplot was generated using the R software's “ggplot2” program, and the heatmap was created using the R software's “pheatmap” tool in the R [9].

### 2.7. Immune Cell Infiltration

We used immunedeconv to evaluate the validity of the immune score assessment results. It is an R software package that includes several recently developed algorithms, such as single-sample gene set enrichment analysis (ssGSEA), ESTIMATE, and EPIC. After benchmarking, each of these algorithms had a distinct advantage. Simultaneously, *SIGLEC15*, *IGIT*, *PDCD1LG2*, *D274*, *AVCR2*, *DCD1*, *TLA4*, and *AG3* genes were chosen as immune checkpoint transcripts, and their expression levels were determined.

### 2.8. Single-Cell Analysis

Tabula Muris is a single-cell transcriptomics platform that contains over 100,000 cells from over 20 different organs and tissues. We investigated the link between the ETNK2 gene expression levels and cell types and tissues in kidney tissue.

### 2.9. Immunohistochemistry (IHC) Analysis Using the Human Protein Atlas (HPA) Database

The HPA database (https://www.proteinatlas.org), an Internet application for determining the protein levels in clinical samples, was used to screen the protein expression levels of hub genes in KIRC tissues.

## 3. Results

### 3.1. Analysis of the ETNK2 Gene Expression

We used the R package (version 3.6.4) to compute the differences in expression patterns between normal and cancerous samples within each tumor. We then performed a nonpaired Wilcoxon rank sum test and a signed-rank test to determine the significance of the differences. We found that the ETNK2 gene was significantly upregulated in 14 tumors, including GBM (tumor: 3.46 ± 1.24, normal: 2.10 ± 1.40, *P*=2.3*e* − 33), GBMLGG (tumor: 3.07 ± 0.99, normal: 2.10 ± 1.40, *P*=2.8*e* − 56), LGG (tumor: 2.95 ± 0.87, normal: 2.10 ± 1.40, *P*=1.5*e* − 38), BRCA (tumor: 4.48 ± 1.52, normal: 3.50 ± 1.13, *P*=2.5*e* − 29), LUAD (tumor: 2.43 ± 1.44, normal: 1.75 ± 0.80, *P*=8.5*e* − 24), LUSC (tumor: 3.63 ± 1.16, normal: 1.75 ± 0.80, *P*=3.5*e* − 103), SKCM (tumor: 4.43 ± 1.35, normal: 3.79 ± 1.09, *P*=1.7*e* − 9), THCA (tumor: 4.50 ± 1.16, normal: 3.31 ± 0.84, *P*=4.9*e* − 58), PAAD (tumor: 2.44 ± 1.07, normal: 1.65 ± 1.42, *P*=5.7*e* − 14), UCS (tumor: 3.88 ± 1.14, normal: 3.73 ± 0.33, *P*=5.4*e* − 3), and All (tumor: −0.97 ± 1.79, normal: −2.51 ± 1.99, *P*=8.8*e* − 15), LAML (tumor: −1.83 ± 2.03, normal: −2.51 ± 1.99, *P*=4.4*e* − 5), PCPG (tumor: 3.29 ± 1.12, normal: 1.31 ± 0.46, *P*=8.4*e* − 3), ACC (tumor: 3.93 ± 2.29, normal: 1.97 ± 1.34, *P*=6.7*e* − 13), and others. At the same time, we observed that the ETNK2 gene was significantly downregulated in 17 tumors, including UCEC (tumor: 2.81 ± 1.35, normal: 3.44 ± 0.70, *P*=0.04), CESC (tumor: 2.50 ± 1.52, normal: 4.08 ± 0.73, *P*=2.7*e* − 5), STES (tumor: 1.25 ± 1.97, normal: 2.27 ± 1.70, *P*=3.4*e* − 29), KIRP (tumor: 3.59 ± 1.13, normal: 5.17 ± 1.71, *P*=1.4*e* − 38), KIPAN (tumor: 3.40 ± 1.43, normal: 5.17 ± 1.71, *P*=1.5*e* − 46), COAD (tumor: 0.23 ± 1.44, normal: 1.56 ± 1.68, *P*=2.0*e* − 32), COADREAD (tumor: 0.39 ± 1.42, normal: 1.54 ± 1.67, *P*=3.7*e* − 31), PRAD (tumor: 2.17 ± 0.92, normal: 3.76 ± 0.51, *P*=9.8*e* − 63), STAD (tumor: 0.81 ± 1.76, normal: 1.31 ± 1.71, *P*=6.8*e* − 5), KIRC (tumor: 3.59 ± 1.35, normal: 5.17 ± 1.71, *P*=2.1*e* − 36), LIHC (tumor: 5.29 ± 1.91, normal: 5.82 ± 1.18, *P*=3.2*e* − 3), WT (tumor: 3.38 ± 0.90, normal: 5.17 ± 1.71, *P*=1.9*e* − 33), BLCA (tumor: 2.81 ± 1.17, normal: 3.25 ± 0.75, *P*=0.04), OV (tumor: 3.10 ± 1.23, normal: 4.59 ± 0.47, *P*=2.5*e* − 33), TGCT (tumor: 4.17 ± 0.74, normal: 7.26 ± 0.67, *P*=2.6*e* − 51), KICH (tumor: 1.11 ± 1.18, normal: 5.17 ± 1.71, *P*=5.3*e* − 31), and CHOL (tumor: 3.12 ± 1.16, normal: 6.33 ± 0.52, *P*=7.8*e* − 6) (Figure 1(a)).

### 3.2. Low ETNK2 Gene Expression Predicts Poor Prognosis in KIRC Patients

We used the Cox function from the R software package (version 3.2-7) survival to investigate the relationship between gene expression and patient prognosis for each cancer type, we employed the Cox function that is included in the R software package survival. Following that, a Cox proportional hazards expression model was developed. Additionally, we conducted a statistical analysis using the log-rank test to determine if the prognosis was significant. Finally, we discovered that the status of patients with KIRC corresponds to their prognosis (Figure 1(b)).

### 3.3. Correlation between the ETNK2 Gene Expression and Immunological Checkpoints in Pan-Cancer

The findings illustrated that the multiple immune checkpoints, including LAG-3, CTLA-4, PD-1, and PD-L1, significantly improved the ETNK2 gene expression in KIRC (Figure 1(c)).

### 3.4. ETNK2 Gene Expression and Survival Analysis in KIRC

Figure 2(a) depicts the findings of a GEPIA analysis of the expression pattern of the ETNK2 gene in tumors and normal tissues. Patients with KIRC with low ETNK2 expression had a poor prognosis (Figure 2(b)). At the same time, the expression and survival analysis confirmed the above trend (Figures 2(c) and 2(d)).

### 3.5. Identification of DEGs

The limma package was used to compare DEGs between the low- and high-ETNK2 expression groups. The volcano plot of DEGs was then shown in Figure 3(a). The gene expression pattern in various tissues is represented by different colors in the heatmap depicting the differential gene expression, each corresponding to a specific tissue.  Figure 3(b) depicts the top 50 upregulated and the top 50 downregulated genes.

### 3.6. Enrichment Analyses

The enrichment of the analysis of DEGs revealed that the ETNK2 gene dysregulation is mostly associated with pathways such as valine, leucine, and isoleucine degradation and tryptophan metabolism and the GO terms such as xenobiotic metabolic and small molecule catabolic process (Figures 3(c) and 3(d)).

### 3.7. Immune Cells Infiltration Analysis

According to the results of ssGSEA, the ETNK2 gene expression is mostly positively corrected with neutrophils and substantially negatively corrected with Th1 cells (Figure 4(a)). The findings of the ESTIMATE algorithm revealed that lowering the ETNK2 gene expression significantly reduced the stromal score and immune score (Figure 4(b)). The EPIC algorithm validated the above immune cell infiltration trend (Figure 4(c)). Changes in immune checkpoint-related genes were also caused by the abnormal expression of the ETNK2 gene (Figure 4(d)).

### 3.8. Single-Cell Analysis of the ETNK2 Gene Expression in Different Cells

The Tabula Muris database was used to determine the relationships between the ETNK2 expression and various cells. The findings revealed that the ETNK2 gene is primarily expressed in cells such as kidney capillary endothelial cells (Figure 5).

### 3.9. IHC Analysis

In this subsequent study, we examined the hub genes protein levels in clinical KIRC tissue samples. The HPA database IHC staining results indicated significantly lower positivity for ETNK2 (Figure 6).

## 4. Discussion

The findings of this study suggest that the ETNK2 mRNA level is a prognosis-related factor in determining the prognosis of KIRC [10]. We found the distinct infiltration levels of various tumor-infiltrating lymphocytes (TILs) are linked to varying levels of ETNK2 expression. Furthermore, patients with KIRC who had decreased expression of the ETNK2 gene had distinct immunosuppressive gene expression profiles.

The ETNK2 gene is located on human chromosome 1q32.1, and the product of this gene is expressed in all human tissues. The ETNK2 enzyme, a member of the choline/ethanolamine kinase family, catalyzes the first step in synthesizing cytidine diphosphate ethanolamine. This enzyme is critical in producing phosphatidylethanolamine, a primary component of cellular membranes [11]. Only a few studies have found a link between ETNK2 and cancer, with one finding claiming that increased CpG methylation in the ETNK2 gene promoter is associated with radiotherapy resistance in laryngeal squamous cell carcinoma [12]. However, the ETNK2 mechanism underlying KIRC is unknown. Huang et al. found a panel of dysregulated metabolic-related genes in KIRC, including ETNK2, *MTHFD2*, *HOGA1*, *GLDC*, *ALDH6A1*, *AGXT2*, and *RRM2* [13]. Our study investigated the role of the ETNK2 gene in KIRC further.

KIRC has long been known to be resistant to chemotherapy, and most patients with this cancer continue to respond poorly to targeted antiangiogenic treatments and immune checkpoint inhibitors [14, 15]. However, it remains unknown if the ETNK2 gene can influence immunotherapy resistance. Therefore, it is worth investigating if the ETNK2 gene is involved in the modulation of the immunological milieu and immune checkpoints in KIRC. TILs in cancer patients' tumor microenvironment (TME) can be used to predict prognosis and immunotherapy efficacy [16, 17]. According to our findings, ETNK2 gene expression levels correlate with the expression levels of certain immune cell subpopulations, including neutrophils, Th17 cells, and Th1 cells. CD8+ T cells are the effector cells used in cancer immunotherapy. Generally, CD8+ T lymphocytes are activated to attack malignant cells via Fas-Fas ligand pathways or perforin-granzyme synthesis [18]. Therefore, additional research must be conducted to identify additional checkpoints. In addition, we investigated the interaction between the ETNK2 gene and genes involved in immune checkpoints; SIGLEC15, IGIT, D274, AVCR2, DCD1, TLA4, AG3, and PDCD1LG2 are the molecules with the strongest association. These findings imply that the ETNK2 gene is linked to immune infiltration in TME and could participate in the immunomodulatory mechanisms of the KIRC.

We found that a dysregulated ETNK2 gene was associated with valine, leucine, and isoleucine degradation and the xenobiotic metabolic process. The cause of metabolic heterogeneity within tumors remains unknown. Furthermore, gene expression could not explain the clustering of metabolic processes. A recent study illustrated that changes in metabolic activity in clear cell RCC are not always linked to changes in the expression of genes encoding metabolic enzymes [19]. This could be due to a noncanonical metabolic flux, gene, and protein expression level differences, or cofactor regulation of enzymatic activities. Certain metabolic changes have a link to the gene expression of metabolic enzymes, such as pyruvate levels and the expression of the *PDHA1* and *LDHA* genes. Lower levels of the PDHA1 and LDHA enzymes involved in pyruvate metabolism may be linked to higher pyruvate levels in malignancies. Therefore, the ETNK2 gene can be a useful biomarker for KIRC related to metabolic activities.

Our research still has potential limitations. Our research is based on the analysis of public databases. Our research analysis was retrospective. Therefore, we need more experimental verification and further multicenter, large sample, and prospective research in the future to prove the mechanism of ETNK2 in KIRC patients and develop more effective treatment strategies.

## 5. Conclusion

We found that the ETNK2 gene has a lower expression level in KIRC and that this expression level is linked to patient survival and the progression of malignancies. The level of ETNK2 gene expression in KIRC tumor tissues was moderately positively linked to the degree to which immune cells such as neutrophils infiltrated the tumor. The ETNK2 gene is a potential treatment target or prognostic indicator for KIRC patients. However, the precise mechanisms through which the ETNK2 gene affects the prognosis of KIRC patients have yet to be thoroughly investigated.

## Figures and Tables

**Figure 1:** (a) Boxplot of the ETNK2 gene in pan-cancer. (b) Forest plot of the survival analysis for the ETNK2 gene in pan-cancer. (c) Heatmap of correlations among immune checkpoints and the ETNK2 gene.

**Figure 2:** (a) Boxplot of the ETNK2 gene expression using the GEPIA database. (b) Kaplan–Meier (K–M) curve of KIRC patients between low- and high-ETNK2 groups using the GEPIA database. (c) Boxplot of the ETNK2 gene expression using the TCGA database. (d) K–M curve of KIRC patients between low- and high-ETNK2 groups using the TCGA database.

**Figure 3:** (a) Volcano plot: the volcano plot is created using the fold change and *P* adjust values. Red, blue, and grey dots represent upregulated, downregulated, and nonsignificant genes, respectively. (b) Heatmap: the differential gene expression is represented using a heatmap, which shows the gene expression patterns in different tissues in different colors. This figure depicts a visualization of the top 50 upregulated and 50 downregulated genes. (c) Functional enrichment: the enriched KEGG signaling pathways. (d) Functional enrichment: the enriched GO term.

**Figure 4:** (a) Pop-plot correlation between the ETNK2 gene expression and immune cell infiltration based on ssGSEA. (b) Pop-plot correlation between the ETNK2 gene expression and ImmuneScore and StromalScore. (c) Boxplot of immune cell infiltration differences between high- and low-ETNK2 expression groups. (d) Boxplot of immune checkpoint differences between high- and low-ETNK2 expression groups.

**Figure 5:** Single-cell analysis of the ETNK2 gene expression: (a) the cells are linked to kidney tissues; (b) the level of the ETNK2 gene expression in brain tissues.

**Figure 6:** Immunohistochemistry analysis of the ETNK2 gene in kidney and KIRC tissue.

## Data Availability

The dataset was downloaded from the UCSC (https://xenabrowser.net/) and the HPA databases (www.proteinatlas.org).
